The article "Impact of the Hydraulic Fracturing on Indoor Radon Concentrations in Ohio: A Multilevel Modeling Approach" was retracted in 2025. Reasons: results that could not be reproduced; errors in the data; unreliable results or conclusions; concerns about the data.

# Impact of the Hydraulic Fracturing on Indoor Radon Concentrations in Ohio: A Multilevel Modeling Approach

**DOI:** 10.3389/fpubh.2019.00076

**Published:** 2019-04-10

**Authors:** Yanqing Xu, Mounika Sajja, Ashok Kumar

**Affiliations:** ^1^Department of Geography and Planning, The University of Toledo, Toledo, OH, United States; ^2^Department of Civil and Environmental Engineering, The University of Toledo, Toledo, OH, United States

**Keywords:** radon, hydraulic fracking, multilevel modeling, GIS, zip code

## Abstract

According to the United States Environmental Protection Agency (U.S. EPA), exposure to radon gas is the second leading cause of lung cancer after smoking. Extant research that has reported that fracking activity increases the radon levels. “Fracking” also known as hydraulic fracturing, which is a technology that is used to extract naturally occurring shale gas from the Marcellus and the Utica shales. Based on the data from the Ohio Radon Information System (ORIS) from 2007 to 2014 in Ohio, this research uses multilevel modeling (MLM) to examine the association between the incidences of hydraulic fracturing and elevated airborne radon levels. The ORIS data include information on 118,421 individual records of households geocoded to zip code areas. Individual records include radon concentrations, device types of the test, and seasons. Euclidean distances between zip code centroid to the 1,162 fracking wells are measured at the zip code level. Two additional zip code variables, namely the population density and urbanicity, are also included as control variables. Multilevel modeling results show that at the zip code level, distance to fracking wells and population density are significant and negative covariate of the radon concentration. By comparing with urban areas, urban clusters, and rural areas are significant which linked to higher radon concentrations. These findings lend support to the effect of hydraulic fracturing in influencing radon concentrations, and promote public policies that need to be geographically adaptable.

## Introduction

Radon is a highly radioactive, inert, and colorless gas. Radon gas occurs by the natural decay of uranium in soil, water, and rocks. The primary source of radon gas in Ohio are soil and “Ohio shale.” According to the United States Environmental Protection Agency (U.S. EPA), long- term exposure to radon causes lung cancer, and there are about 21,000 lung cancer deaths every year in the United States (1). Individuals spend about 90% of their time indoors that exposes them to the radon gas and increases the chances of lung cancer from 3 to 14%. The units of radon gas are pico-curies per liter of air and radon gas levels are expressed in alpha particles (2). The designated action limit of indoor radon gas concentration is 4 pCi/l by the USEPA, and the World Health Organization recommended level is 2.7 pCi/l (2, 3).

Hydraulic fracturing, also known as “fracking” or “hydrofracking” is a technique that creates fractures in the rock formation and stimulates the flow of natural gas. Most Eastern United States have the fracking activity in the Marcellus Shale and fracking is also conducted in the Barnett Shale in Texas (4). In Ohio, shale gas is available in the deposits of Marcellus and Utica shales. The densest deposits of shale in the eastern United States stretches from New York through Pennsylvania, Ohio, and Indiana to Illinois (5). Marcellus shale is known to contain elevated radon levels. A research study found a statistical significance between first-floor radon concentrations and the natural gas wells drilled nearby home locations in the Marcellus shale in Pennsylvania (6). Another reference portrayed the health and environmental risks of fracking, describing how the groundwater gets polluted through fracking and how fracking causes the radioactive gasses to elevate (7). Figure 1 demonstrates the Marcellus and Utica Shale Regions in Ohio (8, 9).

**Figure 1:** Distributions of Marcellus and Utica Shales in Ohio (8, 9).

In this paper, the basic two-level multilevel modeling (MLM) is used to investigate whether there is a relationship between radon and fracking in Ohio. MLM is also known as the hierarchical linear model, random-effect model, variance-components model, or mixed model (10). MLM is multiple regression-based modeling used to predict values of dependent variables at more than one level (11). In the research of human-related subjects, such as public health, MLM is a commonly used method of incorporating individual risk factors and neighborhood characteristics (12). The results in this study show a statistical significance between indoor radon concentrations and fracking. Furthermore, according to the existing research, urban areas have lower radon concentrations when compared to the countryside; i.e., rural areas, as people in cities live upstairs in apartments (13), displaced from the ground from which the radon emanates. The current research continues this line of work to examine the effects of urbanicity on radon concentrations. We expect to see urban cluster and rural areas are related to higher radon concentration by comparing with the urban areas, which can be used to support the conclusions from the existing research.

## Method of Approach

### Variables and Data Sources

The Ohio Radon Information System (ORIS) has been developed and maintained by The University of Toledo, Department of Civil and Environmental Engineering to improve the knowledge of public about indoor radon concentration and is accessible to the public. The system collates radon level data for locations in 1,496 zip codes and encompasses all the 88 counties in Ohio (14). The radon databases posted on the ORIS website consist of five distinct databases: homes database, school database, water database, mitigation database, and tester database (1, 15).

The radon tests conducted by the licensed testers in the homes in Ohio are submitted to the ODH, and then these records are delivered to the Department of Civil and Environmental Engineering at The University of Toledo (UT) (1). For this research, only the observations of the testers database in the homes are used, as licensed testers have initial screening data that are more likely to produce accurate results. The raw testers database passed to the UT has the records in a notepad file. Students process the data in a spreadsheet and the data are checked for accuracy to avoid transcription errors. The final testers database includes information on (1) contractor's license number; (2) contact Name; (3) phone number; (4) street address of the contact; (5) city; (6) county; (7) zip code; (8) radon concentration; (9) room code; (10) device code; (11) test type; (12) start date; (13) completion date; (14) season code; (15) quarter; (16) year in which the measurements were made (1, 15).

Mostly, the radon concentrations in homes are from testing in the basement if a basement is present, or from testing on the first floor otherwise (16). There are various radon measuring devices which the licensed testers use that could be classified as active devices and passive devices (17). Information on various devices and their codes (18) is given in Heydinger et al. (18). The data samples for the radon concentrations in homes are collected throughout the year. The radon tester notes down the start date and the completion date for each home. The information on various seasons and their codes that is helpful for the analysis in this research is given in Heydinger et al. (18). Figure 2 shows the yearly radon concentration records collected from the homes. The total number of records is 118,421, which are all included is our study. The smallest number of records is 8,071 in 2009, while the largest number is 24,861 in 2013.

**Figure 2:** Yearly Indoor Radon Concentration records in Ohio.

Further processing of radon data are done by using ESRI ArcGIS software. To get the county map of Ohio, 2015 TIGER Geodatabase of Ohio has been downloaded from the U.S. 2010 Census Bureau (https://www.census.gov/geo/maps-data/data/tiger-geodatabases.html) by following the steps from a reference handbook (19). After adding the county layer to the ArcMap, NAD 1983 Ohio 17N is used as the appropiate projection in the research. The current radon data file with specific addresses for the years 2007–2014 are then geocoded to points. Figure 1 shows the number of fracking wells in each county of Ohio. From the distribution, most of the fracking wells are located in the eastern Ohio, while Athens County has the highest number of fracking wells. Fulton is the only county with more than 20 fracking wells in the western Ohio.

The fracking wells data which are available from the Ohio Department of Natural Resources website (https://gis.ohiodnr.gov/MapViewer/?config=OilGasWells) contains the shapefile of each county in a downloadable zip file^1^. Not every county has oil and gas wells that are suitable for fracking and geologic shale environment. By using the select attribute tool in the ArcGIS 10.6.1, we obtained the exact fracking locations of the wells by selecting wells that have some form of shale in its underground, geologic environment. In addition, only wells active were chosen (producing, drilling, storage, dry hole with oil, and gas show) and drilled after the year 1999. About 57 counties in Ohio have fracking wells. The distance to the fracking wells was measured as the Euclidean distance to the closest well.

For the definition of urbanicity, this research uses the 2010 Census Urban and Rural Classification (https://www.census.gov/geo/reference/ua/urban-rural-2010.html). The U.S. 2010 Census Bureau defines an urban area on census tracts and census blocks that meets minimum population density requirements. Urbanized areas (UA_s_) (50,000 or more people) and urban clusters (UC_s_) (at least 2,500 and <50,000 people) are two types of urban areas (12, 20). A zip code is classified as (1) urbanized Area, (2) urban cluster or (3) rural if its centroid falls within an Urbanized Area, Urban Cluster or rural area, respectively (21).

### Multilevel Modeling (MLM) Analysis

The main purpose of multilevel model is to predict values of some dependent variable based on a function of predictor variables at more than one level.

The MLM analysis includes 118,421 records of indoor radon concentrations for the years 2007–2014 that are nested in the zip codes. The hierarchical structure of the data has two levels: homes (level 1), zip codes (level 2). Radon concentration is treated as dependent variable in the models. Independent variables include device type, season, distance to fracking wells, population density, and urbanicity. Simple two-level structure that can be seen in the following multilevel modeling, with one predictor variable each at level 1 and level 2^10^:

Level 1 (homes) regression equation:

(1) $$\begin{array}{r} {\text{Y}}_{\text{ij}}={\text{β}}_{0\text{j}}+{\text{β}}_{1\text{j}}{\text{X}}_{\text{ij}}+{\text{e}}_{\text{ij}} \end{array}$$

Y_ij_ refers to the radon concentration for an individual home at Level 1 (subscript i refers to individual case, subscript j refers to the zip code); X_ij_ refers to the Level 1 predictor; β_0j_ refers to the intercept of the dependent variable in zip code j (Level 2); β_1j_ refers to the slope for the relationship in zip code j (Level 2) between the Level 1 predictor and the dependent variable; e_ij_ refers to the random errors of prediction for the Level 1 equation.

Level 2 (zip codes) regression equation:

(2) $$\begin{array}{r} {\text{β}}_{0\text{j}}={\text{γ}}_{00}+{\text{γ}}_{01}{\text{W}}_{\text{j}}+{\text{u}}_{0\text{j}} \end{array}$$

(3) $$\begin{array}{r} {\text{β}}_{1\text{j}}={\text{γ}}_{10}+{\text{u}}_{1\text{j}} \end{array}$$

γ_00_ refers to the overall intercept; W_j_ refers to the Level 2 predictor; γ_01_ refers to the overall regression coefficient; u_0j_ refers to the random error component for the deviation of the intercept of a group from the overall intercept; γ_10_ refers to the overall regression coefficient; u_1j_ refers to the error component for the slope.

The regression analysis is performed by using R software. Table 1 shows the different categories of device types and seasons. For this analysis, device 1 (Continuous Radon Monitor), device 2 (E-PERM), device 3 (Active Charcoal), and device 4 (Pre-Mitigation Level) are four dummy variables that code the five device type categories with the homes tested by other device type as the reference type. There are eight classifications of seasons, while season 8 which is Summer & Fall (Jun–Nov) is treated as the reference category. Our model tested the effect of radon concentrations at both homes and zip code levels; different variables are included to check for significance (22). MLM analysis for the merged data from 2007 to 2014 is conducted in this research.

**Table 1:** Device types and seasons for the radon concentrations from 2007 to 2014.

**Code**	**Season**	**Sample size**	**Percentage %**
1	Fall (Sep–Nov)	25,840	21.82
2	Winter (Dec–Feb)	19,229	16.24
3	Spring (Mar–May)	33,909	28.63
4	Summer (June–Aug)	35,638	30.09
5	Fall & Winter (Sep–Feb)	2,095	1.77
6	Winter & Spring (Dec–May)	311	0.26
7	Spring & Summer (Mar–Aug)	753	0.64
8	Summer & Fall (Jun–Nov)	646	0.55
**DEVICE TYPE**			
1	Continuous Radon Monitor	108,655	91.75
2	E-PERM	2,665	2.25
3	Active Charcoal	5,563	4.70
4	Pre-mitigation Level	1,066	0.90
5	Others	472	0.40

## Results and Discussion

The mean radon concentrations among those tested homes is 5.76 pCi/l, which is higher than the safe levels according to the EPA (4.0 pCi/l) and WHO (2.7 pCi/l) standards. The distribution of radon concentration is shown in Figure 3. Higher overall radon concentration is clustered in the central Ohio. The postal code 43557, which locates in the city of Stryker, OH has the highest radon concentration 141.85 pCi/l. According to Figure 3, distance to shale wells is shorter in the eastern Ohio, while zip codes in the southwest areas are further away from the shale wells. Population density is quite low in the southeast areas, whereas zip codes around Columbus, Cleveland, Cincinnati, and Toledo have the highest population density. Among the 1,162 zip codes, around 2.17% of the areas are classified as urban areas, 69.22% of the areas are classified as urban clusters, while the others are rural areas.

**Figure 3:** Distribution patterns of variables at zip code level: **(A)** Radon Concentration (pCi/l); **(B)** Euclidean Distance to Shale Wells (km); **(C)** Population Density (number of people per square mile); **(D)** Urbanicity.

Table 2 below represents the multilevel modeling regression results for the years 2007–2014, which include 118,421 observations that nested in the 1,162 zip codes in Ohio. In Table 2, Model 1 is the unconditional model with only home-level predictors, model 2 adds the zip-code level variables, and model 3 adds seven dummy variables to code the seven years from 2007 to 2014 (2007 as the reference category). The significance values of coefficients of each variable are tested using a two-tailed *z*-test. The *p*-value ≤ 0.05 indicate that the variables are significant, which means that the effect on radon concentrations is due to the independent variable and not due to random effects. Results for all years provide us the information that homes tested for radon with device Active Charcoal show negative relationship with radon levels by comparing with the other devices in the three models. Continuous Radon Monitor, E-PERM, and Pre-Mitigation Level are not statistically significant. Season 2 Winter (Dec–Feb), Season 3 Spring (Mar–May), Season 6 Winter & Spring (Dec–May), and Season 7 Spring & Summer (Mar–Aug) are negatively associated with radon concentration by comparing with the Summer & Fall (Jun–Nov). Season 1 Fall (Sep–Nov) and Season 5 Fall & Winter (Sep–Feb) are not statistically significant which could be due to the unclear definition of the season. The results of this research prove our hypothesis statement that indoor radon concentrations and fracking in Ohio are related. The closer the distance from homes to shale wells, the higher the radon concentrations. Population density is negative associated with radon concentration. Furthermore, by comparing with the urban areas, urban clusters and rural areas tend to have higher radon concentrations. Those results can be explained that people living in the urban areas are more likely to live in apartments, which displaced from the ground from where the radon emanates. Based on the AIC values, Model 3 is preferred.

**Table 2:** Multilevel modeling for radon concentrations from 2007 to 2014.

	**Model 1**	**Model 2**	**Model 3**
**HOME-LEVEL VARIABLES**			
Device 1	0.234	0.219	0.282
Device 2	0.686	0.673	0.758
Device 3	−1.493^**^	−1.500^**^	−1.500^**^
Device 4	0.575	0.554	0.974
Season 1	0.399	0.400	0.493
Season 2	−1.948^***^	−1.948^***^	−1.823^***^
Season 3	−1.449^***^	−1.447^***^	−1.285^**^
Season 4	−0.918^*^	−0.917^*^	−0.764
Season 5	0.441	0.443	0.804
Season 6	−3.111^***^	−3.105^***^	−2.715^***^
Season 7	−2.747^***^	−2.729^***^	−2.334^***^
**ZIP-CODE LEVEL VARIABLES**			
Distance to wells		−0.821^**^	−0.841^**^
Population density		−0.0004^***^	−0.0004^***^
Urban clusters		1.031^**^	0.992^*^
Rural		1.411**	1.389*
**YEARS**			
2008			0.214
2009			0.747^***^
2010			0.879^***^
2011			0.403^**^
2012			1.025^***^
2013			0.114
2014			0.109
*AIC*	*875601.3*	*875586.7*	*875460.5*

*Sample size: 118,421 observations tested in 1,162 zip codes*.

*** p ≤ 0.001,

** p ≤ 0.01,

* *p ≤ 0.05 (two-tailed tests)*.

Table 3 shows the regression analysis for individual years. Results for the year 2014 provide us the information that homes tested for radon with devices Continuous Radon Monitor, E-PERM, Active Charcoal, and Pre-Mitigation Level show no significant relationships with radon levels by comparing with other devices. Season Fall (Sep–Nov) is slightly positively associated with radon concentration by comparing with the Summer & Fall (Jun–Nov). Nearest distances to the fracking wells calculated for this year prove that there is a slightly negative relationship between fracking and indoor radon levels. Considering the regression results for the year 2013, homes tested for radon with different devices show the same pattern as the year 2014. In addition, radon tested in different seasons shows no significant correlation with radon concentration by comparing with Summer & Fall (Jun–Nov). Population density is also significant which provides us with the information that the larger the population density, the smaller the radon concentration. However, there is no relationship between the distances to the fracking wells and the radon levels. In view of the regression results for the year 2012, homes tested for radon with different device types and seasons show the same pattern as the year 2013. Population density is negatively associated with radon concentration. The distance to fracking wells show robust statistical significance, the shorter the distance from the fracking locations to the homes, the higher the radon concentrations. For the year 2011, homes tested for radon with different devices are not statistically significant when compared to those homes tested with other devices. Moreover, radon levels tested in the Season Fall (Sep–Nov) is positively associated with indoor radon levels by comparing with the Summer & Fall (Jun–Nov). Both distance to shale wells and population density are strongly negatively associated with radon concentrations, which show the same pattern as the year 2012.

**Table 3:** Multilevel modeling for radon concentrations for different years.

	**2007 (*N* = 11,419)**	**2008 (*N* = 11,749)**	**2009 (*N* = 8,071)**	**2010 (*N* = 8,193)**
**HOME-LEVEL VARIABLES**				
Device 1	−0.240	1.435	0.067	−0.458
Device 2	−1.083	−0.442	0.592	−0.379
Device 3	−0.794	−0.340	−2.706^***^	0.095
Device 4	0.454			
Season 1	1.327	2.434	−0.764	−0.518
Season 2	−1.027	−1.108	−3.175^***^	−3.223
Season 3	−0.379	−0.608	−2.351^***^	−2.587
Season 4	−0.045	0.475	−1.177^**^	−2.868
Season 5	0.058		0.520	
Season 6	−1.433			
Season 7	0.917			
**ZIP-CODE LEVEL VARIABLES**				
Distance to wells	−0.904^*^	−0.635^*^	−0.861^*^	−1.091^**^
Population density	−0.0003^*^	−0.0002^*^	−0.0005^***^	−0.0004^**^
Urban clusters	0.219	−0.322	−0.240	−0.308
Rural	−0.025	0.097	0.705	0.0471
*AIC*	*78023.33*	*93968.9*	*55547.59*	*58241.73*
	**2011 (*****N*** **=** **13,777)**	**2012 (*****N*** **=** **17,405)**	**2013 (*****N*** **=** **24,861)**	**2014 (*****N*** **=** **22,946)**
**HOME-LEVEL VARIABLES**				
Device 1	−0.729	0.998	1.750	1.858
Device 2	0.068	−0.026	2.270	3.068
Device 3	−1.508	0.188	−0.356	−0.475
Device 4				
Season 1	3.540^**^	4.820	3.766	1.685^*^
Season 2	1.233	1.967	2.263	−0.207
Season 3	1.280	3.084	2.851	−0.056
Season 4	1.652	3.160	3.318	0.628
Season 5	1.146	2.877	4.968	−3.699
Season 6			0.904	1.533
Season 7		2.488	1.799	−1.332
**ZIP-CODE LEVEL VARIABLES**				
Distance to wells	−1.587^**^	−0.7944^**^	−0.468	−0.878^*^
Population density	−0.001^***^	−0.0003^***^	−0.0004^***^	−0.0005^***^
Urban clusters	1.283	−0.984	−1.109	−0.012
Rural	1.187	−1.306	−0.825	0.170
*AIC*	*99200.79*	*130581.4*	*179878.2*	*174456.5*

*** p ≤ 0.001,

** p ≤ 0.01,

* *p ≤ 0.05 (two–tailed tests)*.

The results presented for the year 2010 do not show any statistical significance for device types and seasons. There is negative relationship between the distance to fracking wells and indoor radon levels. The relationship between population density and radon concentration also show the same pattern. Considering the MLM regression results for the year 2009, device Active Charcoal is strongly negatively associated with radon concentrations by comparing with the other devices tested for homes. Radon concentrations tested with the Continuous Radon Monitor, E-PERM and Pre-Mitigation Level devices do not show significance. On the other hand, radon levels tested in the seasons Winter (Dec-Feb), Spring (Mar-May), and Summer (June-Aug) show statistically significance with radon concentration by comparing with the Summer & Fall (Jun–Nov). The AIC value for the model in 2009 demonstrates that it is the best model by comparing with models tested in the other years. Results for the year 2008 and 2007 provide us the information that homes tested for radon with different devices types show no significant relationship with radon levels by comparing with the other devices. Different seasons do not show statistical significance. Nearest distances calculated for the year 2008 and 2007 demonstrate that there is a weak correlation between fracking and indoor radon levels. Population density also shows slightly significance of the effects of radon level. Urban clusters and rural clusters do not show any significant differences compared to urbanized areas for all models for individual years.

## Concluding Comments

Based on the radon data from 2007 to 2014 in Ohio, this research examines the associations between the nearest distance to fracking wells and household radon levels after controlling for individual radon related risk factors. The independent variables demonstrate inconsistent statistical significance on the radon concentration among different years from 2007 to 2014, which suggest that the radon concentration data are not distributed equivalently throughout Ohio. The limitation of the study should be kept in mind when interpreting study findings. The most important concern is the data. The measurement of radon concentration relied on self-reported devices and thus was subject to response bias.

The statistical results interpret that there is a strong correlation between indoor radon concentrations and hydraulic fracturing in Ohio. The licensed testers provide the name of the device used and the season code variables considered. Distance to the fracking well locations from the homes, population density, and urbanicity are included as zip code level variables. For the first time, two-level MLM analysis is used for this type of research. The MLM analysis results provide us with information that among the variables used: (i) nearest distance of homes from the fracking well locations at the zip code level is significant in all the years; and (ii) population density and different urbanization levels show strong significance with radon concentrations.

## Author Contributions

All authors listed have made a substantial, direct and intellectual contribution to the work, and approved it for publication.

### Conflict of Interest Statement

The authors declare that the research was conducted in the absence of any commercial or financial relationships that could be construed as a potential conflict of interest.

## Footnotes

^1^ODNR Oilgas Wells. https://gis.ohiodnr.gov/MapViewer/?config=OilGasWells.
